The article "High-Affinity Naloxone Binding to Filamin A Prevents Mu Opioid Receptor–Gs Coupling Underlying Opioid Tolerance and Dependence" was retracted in 2022. Reasons: duplicated images; concerns about the data; concerns about the images.

# High-Affinity Naloxone Binding to Filamin A Prevents Mu Opioid Receptor–Gs Coupling Underlying Opioid Tolerance and Dependence

**DOI:** 10.1371/journal.pone.0001554

**Published:** 2008-02-06

**Authors:** Hoau-Yan Wang, Maya Frankfurt, Lindsay H. Burns

**Affiliations:** 1 Department of Physiology and Pharmacology, City University of New York Medical School, New York, New York, United States of America; 2 Pain Therapeutics, Inc., San Mateo, California, United States of America; University of California, Berkeley, United States of America

## Abstract

Ultra-low-dose opioid antagonists enhance opioid analgesia and reduce analgesic tolerance and dependence by preventing a G protein coupling switch (Gi/o to Gs) by the mu opioid receptor (MOR), although the binding site of such ultra-low-dose opioid antagonists was previously unknown. Here we show that with approximately 200-fold higher affinity than for the mu opioid receptor, naloxone binds a pentapeptide segment of the scaffolding protein filamin A, known to interact with the mu opioid receptor, to disrupt its chronic opioid-induced Gs coupling. Naloxone binding to filamin A is demonstrated by the absence of [^3^H]-and FITC-naloxone binding in the melanoma M2 cell line that does not contain filamin or MOR, contrasting with strong [^3^H]naloxone binding to its filamin A-transfected subclone A7 or to immunopurified filamin A. Naloxone binding to A7 cells was displaced by naltrexone but not by morphine, indicating a target distinct from opioid receptors and perhaps unique to naloxone and its analogs. The intracellular location of this binding site was confirmed by FITC-NLX binding in intact A7 cells. Overlapping peptide fragments from c-terminal filamin A revealed filamin A_2561-2565_ as the binding site, and an alanine scan of this pentapeptide revealed an essential mid-point lysine. Finally, in organotypic striatal slice cultures, peptide fragments containing filamin A_2561-2565_ abolished the prevention by 10 pM naloxone of both the chronic morphine-induced mu opioid receptor–Gs coupling and the downstream cAMP excitatory signal. These results establish filamin A as the target for ultra-low-dose opioid antagonists previously shown to enhance opioid analgesia and to prevent opioid tolerance and dependence.

## Introduction

Ultra-low-dose opioid antagonists have been shown to enhance opioid analgesia and attenuate tolerance and dependence, with a mechanism long hypothesized as a blockade of excitatory signaling opioid receptors [1]–[4]. Ultra-low-dose opioid antagonists can also reverse hyperalgesia caused by acute, low-dose opioids to produce analgesia [5]. Additionally, ultra-low-dose naltrexone has recently been shown to attenuate opioid reward or addictive properties in conditioned place preference [6] and self-administration and reinstatement paradigms [7]. In a recent clarification of the mechanism of action of ultra-low-dose opioid antagonists, we showed that co-treatment with 10 ng/kg naloxone (NLX) prevented a chronic morphine-induced, Gi/o-to-Gs switch in G protein coupling by the mu opioid receptor (MOR) as well as a coincident interaction of the Gβγ dimer with adenylyl cyclase II and IV [4]. While opioid receptors preferentially bind Gi and Go proteins to inhibit adenylyl cyclase [8], chronic morphine induces MOR–Gs coupling [4], [9]. Although Chakrabarti et al (2005) also demonstrated some MOR–Gs coupling in the opioid naïve state while we did not, we believe this difference may be due to their use of non-immobilized anti-Gα antibodies producing some background binding by Fc receptors. First postulated as the sole mediator of excitatory effects of opiates [10], the Gβγ interacting with adenylyl cyclases originates from the Gs protein coupling to MOR and not from MOR's native G proteins [11].

Ultra-low-dose opioid antagonists were initially thought to preferentially bind a subset of MORs [1], and a Gs-coupling MOR subpopulation was again recently proposed [9]. While it is difficult to estimate the relative proportion of MORs signaling via Gs versus Gi/o during tolerance, it seemed unlikely that the ultra-low doses of NLX or naltrexone influencing opioid agonist effects would be sufficient to selectively antagonize such a subpopulation. Based on saturation binding studies [12], which incorporate NLX's affinity to MOR, we estimate receptor occupancy of 10 ng/kg NLX as no more than 1%. More importantly, our co-immunoprecipitation data showed that ultra-low-dose NLX co-treatment reduces MOR–Gs coupling while *restoring* levels of coupling to MOR's native Gi/o proteins; further, in spinal cord of co-treated rats, MOR–Gi/o coupling levels greatly surpassed those of opioid-naïve rats [4]. If NLX were selectively antagonizing a subpopulation of “Gs-coupled” MORs, coupling to native G proteins would likely be unaffected.

Since NLX prevents MOR–Gs coupling at concentrations well below its affinity for MOR and by influencing the coupling behavior of MORs, we considered proteins that interact with MOR and MOR-associated G proteins as the most likely targets, particularly those able to interact with multiple MORs. We first examined proteins that co-immunoprecipitated with MOR during activation. We identified a 300-kDa protein co-immunoprecipitating with MOR as FLNA and then demonstrated specific, high-affinity binding by NLX to FLNA. Best known for cross-linking cytoplasmic actin into dynamic scaffolds to control cell motility, filamins are large cytoplasmic proteins increasingly found to regulate cell signaling by interacting with over 30 different receptors and signaling molecules [13], [14], including MOR [15]. We deduced the precise binding site on FLNA by using overlapping peptides within the c-terminal, since c-terminal FLNA was shown to interact with MOR using a yeast-two hybrid [15]. To assess the functional significance of this high-affinity interaction, we used peptide fragments containing the binding site to prevent NLX from binding full-length FLNA in organotypic striatal slice cultures. Our findings suggest that FLNA interacts with ultra-low-dose NLX and naltrexone to prevent chronic morphine-induced MOR–Gs coupling, possibly by preventing a critical MOR–FLNA interaction. This high-affinity binding site in c-terminal FLNA therefore appears to underlie the paradoxical enhancement of opioid analgesia and prevention of analgesic tolerance and dependence by ultra-low-dose opioid antagonists. In identifying the binding site though which ultra-low-dose opioid antagonists prevent MOR–Gs coupling, our data also reveal an important regulation of MOR–G protein coupling by filamin A.

## Results

### Identification of NLX-binding protein in MOR immunoprecipitates

In previous co-immunoprecipitation experiments of MOR and G proteins, we noted a protein with molecular weight at approximately 300-KDa in Gαi/o immunoprecipitates in an amount that closely paralleled the amount of MORs in these immunoprecipitates, suggesting a functional interaction. A battery of antibodies against various cytoskeletal proteins, preliminarily identified this protein that co-immunoprecipitated with MORs and their associated G proteins as FLNA. Using striatal tissue of rats treated chronically with vehicle, morphine, ultra-low-dose NLX or morphine+ultra-low-dose NLX, we performed a two-tiered co-immunoprecipitation with anti-Gα followed by anti-MOR antibodies. The final probing with a specific anti-FLNA antibody showed that FLNA associates with Go-coupled MOR and not with Gs-coupled MOR (Fig. 1 A,B). These blots also demonstrate the morphine-induced G protein coupling switch by MOR and its attenuation by co-treatment with ultra-low-dose NLX. The blots were stripped and re-probed with antibodies to MAP_1B_ and yaotio to illustrate the absence of these cytoskeletal proteins in these immunoprecipitates (Fig. 1C). The exclusive presence of FLNA in the MOR/Go complexes led us to hypothesize that FLNA is the target through which ultra-low-dose NLX blocks the chronic morphine-induced switch from normal MOR–Gi/o coupling to Gs coupling.

**Figure 1:** FLNA associates with Go-coupled MORs and not Gs-coupled MORs. Neuronal membranes were prepared from striata of rats chronically treated with vehicle, morphine, or ultra-low-dose NLX alone or combined with morphine. After stimulation by *in vitro* morphine or not, membranes were solubilized and immunoprecipitated first with immobilized anti-Gα. Anti-Gα immunoprecipitates were then immunoprecipitated with immobilized anti-MOR before final Western blot detection with anti-FLNA. Densitometric quantitation (*B*) of Western blots of both MOR in the second immunoprecipitate and FLNA in the final (*A*) demonstrates that FLNA is associated with MORs coupling to Go but not MORs coupling to Gs. These blots and their quantitation also show that NLX co-treatment prevented the chronic morphine-induced Go-to-Gs coupling switch. Solid bars indicate basal coupling, and hatched bars indicate coupling after receptor stimulation by* in vitro* morphine. *n* = 4. *p<0.05, **p<0.01 compared to respective basal coupling level. # p<0.01 compared to respective value in vehicle or morphine+NLX groups. Blots were stripped and re-probed with antibodies to yaotio, MAP2, H-neurofilament and MAP1B (*C*).

### NLX binding in FLNA-expressing cells and affinity measurement

To validate the binding of NLX to FLNA, we assessed binding of [^3^H]NLX to membranes prepared from the human melanoma cell line M2 that lacks filamin and to membranes from its FLNA-transfected subclone A7. We first confirmed FLNA expression in A7 cells and absence in M2 cells by Western blotting using a specific anti-FLNA antibody (Table 1). FLNA was also detected in the human neuroblastoma SK-N-MC cell line and in rat cortical membranes (Table 1). Importantly, [^3^H]NLX bound to A7 membranes and this binding was robustly displaced by naltrexone but not by morphine, illustrating that NLX and naltrexone bind to a novel site distinct from MOR (Fig 2A). Negligible [^3^H]DAMGO binding to A7 cells suggested that these cells (and presumably their M2 parent line) do not express MORs (Fig. 2B). Finally, the filamin-deficient M2 cells do not express molecules that bind [^3^H]NLX (Fig. 2C).

**Figure 2:** NLX target is distinct from MOR but also bound by naltrexone. *A,* Naltrexone but not morphine markedly reduced [^3^H]NLX binding in FLNA-expressing A7 membranes. *n* = 6. *B,* The absence of [^3^H]DAMGO binding using twice the amount of A7 membranes shows these lines do not express MOR. *n* = 4. *C,* Parent M2 melanoma cells do not express NLX targets. *n* = 4. * p<0.05 compared to control.

**Table 1:** FLNA expression (Optical intensity of Western blot bands, arbitrary units)

	A7 cells	M2 cells	SK-N-MC cells	Rat cortex
15 µg	825.8±69.6	0±0	351.3±63.9	230.3±29.4
30 µg	2454.8±259.9	0±0	983.8±89.0	664.8±67

Solubilized proteins (15 or 30 µg) from membrane preparations were size-fractioned by 7.5% SDS-PAGE and electrophorectically transferred onto nitrocellulose for Western blotting using specific anti-FLNA antibodies. n = 4.

In an affinity assessment, a competition (displacement) curve for the inhibition of [^3^H]NLX binding to A7 cell membranes was performed using 16 concentrations of naltrexone. Analysis by nonlinear regression showed two saturable sites (R^2^ = 0.9788) with an IC_50_-H of 3.94 picomolar and an IC_50_-L of 834 picomolar (Fig. 3).

**Figure 3:** NLX binds A7 membranes with picomolar affinity. A competition (displacement) curve for the inhibition of [^3^H]NLX binding by naltrexone to membranes from FLNA-expressing A7 cells shows two affinity states with IC_50_-H of 3.94 picomolar and IC_50_-L of 834 picomolar. A nonlinear curve-fit analysis was performed using a competition equation that assumed two saturable sites for the naltrexone curve comprising of 16 concentrations ranging from 0.1 pM to 1 µM. Data are derived from 6 experiments each using a different set of A7 cells.

### Precise NLX binding site determined using overlapping peptides

To deduce the precise binding domain within FLNA where NLX binds, several overlapping peptide sequences derived from the carboxy-terminus where FLNA intersects with synaptic membranes were used to absorb [^3^H]NLX. Both FLNA_2556–2565_ and FLNA_2561–2570_ markedly attenuated [^3^H]NLX binding to A7 cell membranes and to purified human FLNA (Fig. 4). This result was confirmed using FLNA purified from FLNA- and MOR-expressing SK-N-MC cells. At 500 pM concentration, [^3^H]NLX binds to immunoaffinity-purified FLNA in the presence or absence of irreversible MOR antagonist, β-FNA. These data together suggest that NLX binds with high affinity to FLNA with the binding site located at FLNA_2561–2565_.

**Figure 4:** FLNA_2561–2565_ is the binding site for [^3^H]NLX. A7 cell membranes or purified FLNA was incubated with [^3^H]NLX in the presence of various overlapping FLNA c-terminal peptide fragments. Peptides containing FLNA_2561–2565_ markedly reduced [^3^H]NLX binding to A7 membranes (*A*) and to purified FLNA (*B, C*). The reduction of [^3^H]NLX binding to purified FLNA was not affected by the presence of the irreversible MOR antagonist β-FNA (*C*). *n* = 6. * p<0.01 compared to vehicle.

### Confirmation of pentapeptide binding and alanine scan

To confirm that FLNA_2561–2565_ binds NLX and to deduce the critical amino acid(s) within the NLX interacting FLNA_2561–2565_ region, we generated 4 alterations of FLNA_2561–2565_ each with 1 amino acid replaced by alanine (alanine scan). Using FLNA_2561–2565_ and the alanine-replaced pentapeptides to compete with [^3^H]NLX binding to FLNA in A7 cell membranes, we show that the lysine residue at FLNA_2663_ is critical to the NLX–FLNA interaction. While the FLNA_2561–2565_ displacement of [^3^H]NLX binding was only slightly attenuated by alanine substitutions at the first, fourth and fifth amino acid residues, substitution of the lysine completely prevented it (Fig. 5). The notion that NLX binds to the extreme carboxyl terminus of FLNA that tethers to the internal potion of cell membranes is supported by our data illustrating that FLNA_2561–2565 _(VAKGL) prevented the [^3^H]- and FITC-NLX labeling that localized internally in intact A7 but not M2 cells (Fig. 6). This labeling occurred without membrane permeabilization, indicating that NLX can easily penetrate cell membranes to access FLNA.

**Figure 5:** Mid-point lysine of FLNA_2561–2565_ is critical for NLX binding. An alanine scan of the FLNA_2561–2565_ pentapeptide (VAKGL) shows that residue of FLNA_2561–2565_ is critical for NLX binding. All other individual alanine substitutions only mildly attenuated [^3^H]NLX binding to FLNA in A7 membranes. *n* = 6. * p<0.01 compared to vehicle.

**Figure 6:** [^3^H]- and FITC-NLX binding to intact A7 cells is blocked by FLNA_2561-2565_. Intact A7 and M2 cells were incubated with 0.5 nM [^3^H]NLX or 10 nM FITC-NLX in the presence or absence of 10 nM VAKGL or VAAGL. [^3^H]NLX bound to A7 but not to M2 cells and VAKGL markedly reduced this binding to A7 cells (*A*). Likewise, FITC-NLX labelled A7 (*B.I*) but not M2 cells (*B.II*), and co-treatment with VAKGL (*B.III*) but not VAAGL (*B.IV*) abolished this FITC-NLX labelling in A7 cells (*B*). *n* = 4. * p<0.01 compared to vehicle.

### Peptide binding site interferes with NLX's prevention of MOR–Gs coupling induced by chronic morphine

To confirm that NLX binding to FLNA prevents the chronic morphine-induced Gi/o-to-Gs coupling switch, we utilized organotypic rat brain striatal slice cultures. We previously showed that *in vivo* chronic morphine induced a switch to MOR–Gs coupling in rat striatum, periaqueductal gray and dorsal spinal cord from Gi or Go coupling in these latter two regions but from an exclusive Go coupling in striatum [4]. To mimic the *in vivo* chronic morphine treatment and resulting opioid tolerance in that study, rat striatal slices were treated for 7 days twice daily for 1 hr with 100 µM morphine in serum-free culture medium. This morphine treatment induced a robust Go-to-Gs coupling switch, similar to that previously observed following *in vivo* chronic morphine, that was also similarly blocked by co-treatment with ultra-low-dose (10 pM) NLX (Fig. 7). The addition of FLNA_2561–2570_ but not FLNA_2550–2560_ or FLNA_2566–2575_ abolished NLX's prevention of the Go-to-Gs coupling switch, presumably by preventing NLX from binding FLNA in the tissue (Fig. 7). Densitometric quantitations of blots from slices treated with NLX or FLNA peptides alone did not differ from those of vehicle and are omitted from Fig. 7B for simplification.

**Figure 7:** FLNA_2561-2565_ blocks 10 pM NLX's prevention of the chronic morphine-induced Go-to-Gs coupling switch. Striatal slices were chronically treated with vehicle, morphine, NLX, morphine+NLX, or with one of the three FLNA peptides alone or in combination with morphine+NLX. Coupling between MOR and Gs/Go proteins was assessed by Western blot (*A*) and analyzed by densitometric scanning (*B*). Chronic morphine exposure caused a Go-to-Gs coupling switch that was blocked by NLX co-treatment. NLX's suppression of this coupling switch was blocked by FLNA_2561-2570_ but not by FLNA_2566–2575_ or FLNA_2550–2560_, illustrating that NLX's protective effect occurs via its binding to FLNA within FLNA_2561–2570_. Solid bars indicate basal coupling; hatched bars indicate coupling after *in vitro* morphine stimulation. *n* = 6. *p<0.01 compared to Kreb's Ringer; +p<0.01 compared to morphine; #p<0.01 compared to morphine+NLX.

Consistent with the G protein coupling switch, morphine treatment also increased basal cAMP levels, caused DAMGO to stimulate cAMP production, and attenuated the DAMGO-mediated reduction in forskolin-stimulated cAMP accumulation (Fig. 8). As with the coupling switch, the addition of FLNA_2561–2570_ but not FLNA_2550–2560_ or FLNA_2566–2575_ abolished NLX's prevention of these cAMP indices of morphine tolerance. Treatment with NLX or FLNA peptides alone did not alter cAMP levels from those of vehicle (data not shown). These data together suggest that ultra-low-dose NLX prevents analgesic tolerance in response to chronic morphine by binding to a specific region of FLNA.

**Figure 8:** FLNA_2561–2565_ blocks 10 pM NLX's prevention of chronic morphine-induced cAMP accumulation. After chronic treatments, slices were stimulated with DAMGO, forskolin or DAMGO+forskolin before solubilizing tissues and measuring cAMP levels. In accordance with the Go-to-Gs coupling switch, chronic morphine increased basal cAMP production by 24%, caused DAMGO to stimulate basal cAMP production, and reduced the DAMGO-mediated inhibition of the forskolin effect from 35% in vehicle/NLX groups to 7%. NLX co-treatment blocked these morphine-induced effects, and the protective effect of NLX was blocked by FLNA_2561–2570_ but not by FLNA_2566–2575_ or FLNA_2550–2560_, again demonstrating that NLX's protection occurs through binding to FLNA within FLNA_2561–2570_. *n* = 4. *p<0.01 compared to forskolin alone. +p<0.01 compared to vehicle. ##p<0.05, #p<0.01 compared to basal level.

## Discussion

We have identified a high-affinity binding site for NLX in the carboxyl-terminal region of the scaffolding protein FLNA that appears to mediate ultra-low-dose NLX's prevention of the chronic opioid-induced G protein coupling switch by MOR. This finding further elucidates the mechanism of action of certain ultra-low-dose opioid antagonists in enhancing opioid analgesia and preventing opioid tolerance and dependence [4]. We measure the binding affinity of NLX or naltrexone to FLNA in cell membranes as 4 picomolar, i.e. approximately 200-fold higher than their binding affinity for MOR [16], [17]. To our knowledge, this is the first demonstration of picomolar binding by a psychoactive compound that is not to a cell surface receptor. NLX binds FLNA tightly with critical involvement of a 5-amino acid segment that is intracellular but near its c-terminal transmembrane domain.

The presence of FLNA in MOR signalplex in native brain tissues demonstrated here by co-immunoprecipitation agrees with previous data using yeast-two hybrid and co-transfection methods [15]. The dependence of [^3^H]NLX binding on FLNA expression in cell lines, the absence of MOR in these cell lines, and the displacement by naltrexone but not morphine clarified FLNA as a novel target for NLX and naltrexone. The interaction was confirmed using immunopurified FLNA from A7 or SK-N-MC cells. Since FLNA_2556–2565_ and FLNA_2561–2570_ both markedly reduced [^3^H]NLX binding to A7 membranes or to purified FLNA proteins, we assumed that FLNA_2561–2565_, within the 24^th^ repeat, is the NLX-binding site on FLNA. We confirmed FLNA_2561–2565 _as the binding site by showing NLX binding to this pentapeptide_, _and an alanine scan revealed that the lysine at FLNA_2563_ is critical for binding. We cannot easily explain a modest enhancement in NLX binding caused by FLNA_2575–2583_, but this could be the result of reducing steric constraints around the NLX binding site on FLNA. Our demonstration that FLNA_2561–2565_ (VAKGL) but not VAAGL abolished [^3^H]- and FITC-NLX binding to intact A7 cells again confirmed that this pentapeptide is a NLX binding site and demonstrated that NLX can access this intracellular target. Finally, the blockade of NLX's protective effects on both Gs coupling and cAMP accumulation by peptides containing FLNA_2561–2565_ provides evidence that ultra-low-dose NLX may block MOR–Gs coupling and associated opioid tolerance and dependence by binding to FLNA at approximately FLNA_2561–2565_. Although MOR desensitization, i.e. the decrease in coupling to native G proteins, is more commonly thought to underlie opioid tolerance and dependence [18], [19] than a switch to Gs coupling, our present data indicate that a decrease in MOR efficacy can not alone mediate chronic opioid effects. Specifically, the increase in cAMP accumulation caused by DAMGO without forskolin following chronic morphine treatment illustrates that MOR has not merely desensitized, losing its ability to inhibit cAMP production, but that its stimulation actually augments cAMP production.

The detection of FLNA in immunoprecipitates containing Go-coupled MOR and not Gs-coupled MOR appears counterintuitive since NLX prevents MOR–Gs coupling via a tight binding to FLNA. We propose that repeated MOR stimulation may force a particular conformation of the MOR-FLNA complex that weakens the entire signalplex. MOR may subsequently release from both its native G protein and from FLNA itself leading to association with Gs without FLNA in the complex. By binding to FLNA, NLX could block this particular MOR–FLNA interaction and stabilize the MOR-FLNA-G protein complexes, thereby reducing the morphine-induced release of MORs and their subsequent coupling with Gs in response to receptor stimulation. MOR and FLNA might be forced into an altered conformation or interaction during opioid tolerance by proteins involved in MOR recycling and internalization such as β-arrestins [20]. Additionally, as exogenous GM1 ganglioside has been shown to mimick opioid tolerance *in vitro* [21] and since blocking GM1 ganglioside via cholera toxin B subunit also blocks the excitatory effects of opiates *in vitro* [22] and *in vivo* [23], GM1 ganglioside may also influence MOR–FLNA interactions. Interestingly, although we observed FLNA in MOR signalplexes containing Go proteins in native brain tissue, the prior data in co-transfected cells indicates that FLNA is not required for the native coupling state of MOR; in fact, its absence actually enhances MOR function [15].

This prior study by Onoprishvili et al., the first to show that FLNA interacts with the c-terminal of MOR, proposed a role for FLNA in receptor regulation and trafficking [15]. The authors reported that MOR functioned normally in cells lacking FLNA, but that the agonist DAMGO was unable to desensitize MOR, as measured by the decreased ability of DAMGO to inhibit forskolin-mediated cAMP accumulation following prolonged DAMGO exposure. In agreement, our present slice culture data show that ultra-low-dose NLX, by binding to FLNA, prevents this morphine-induced desensitization measure, as well as the upstream MOR–Gs coupling that we previously showed to underlie tolerance and dependence *in vivo* [4]. Rather than desensitization, Onoprishvili et al. actually noted *enhanced* inhibition by DAMGO of cAMP accumulation in cells lacking FLNA [15], a finding that also agrees with the idea that in signaling complexes that do not contain FLNA, MOR does not release from its Gi/o protein to interact with Gs. This increased Gi/o recruitment leading to heightened DAMGO-induced cAMP inhibition also concurs nicely with the increased Gi/o coupling we previously observed in spinal cord of animals treated with morphine+ultra-low-dose NLX [4], as well as with the enhanced analgesia that follows these co-treatments [2].

It is possible that the ultra-low-dose opioid antagonist attenuation of opioid addictive properties [6], [7] may also be mediated by this high-affinity binding to FLNA. While the enhancement of opioid analgesia and reduction of analgesic tolerance is “paradoxical,” and occurs only at “ultra-low” doses of NLX and naltrexone (since higher doses of these opioid antagonists also antagonize opioid receptors), the attenuation of rewarding or addictive properties of opioids by ultra-low-dose naltrexone is not paradoxical. Hence, one would expect a continuous suppression of reward as increasing doses of naltrexone are combined with the opioid. Yet, in the conditioned place preference paradigm, while both ultra-low (0.03 and 0.3 ng/kg) and higher (30 ng/kg) naltrexone doses blocked the acute rewarding effects of oxycodone, an interim dose (3 ng/kg) was without effect [6]. Similarly, in a self-administration paradigm, while co-self-administering 10 or 1 pg/kg/infusion both attenuated measures of reinstatement when oxycodone was not available, only the lower dose altered oxycodone's rewarding potency during self-administration [7]. The blunting of opioid rewarding effects by ultra-low-dose naltrexone first suggests that Gs coupling by MOR may contribute to the rewarding or addictive properties of opioids, possibly by cAMP activation of PKA and subsequent CREB phosphorylation. However, opioid inhibitory effects, such as the proposed disinhibition of VTA dopamine neurons via inhibition of GABA interneurons [24], may also contribute to opioid reward. The loss of effect at intermediate naltrexone doses may indicate such complexities of the neural mechanisms contributing to opioid reward and addiction. Alternatively, the fact that the attenuation of rewarding effects is diminished as the naltrexone dose increases could also suggest an upper limit of an effective ultra-low dose range for disrupting the FLNA–MOR interaction and consequent MOR–Gs signaling.

In summary, here we identify a specific c-terminal region of FLNA as the high-affinity binding site of NLX and naltrexone in their suppression of MOR signaling alterations that result from chronic opioid treatment. This work therefore provides a molecular target for ultra-low-dose NLX through which ultra-low-dose opioid antagonists enhance opioid analgesia and decrease opioid tolerance and dependence. We propose that repeated MOR stimulation leads to a particular conformation of MOR–FLNA that weakens Gi/o–MOR–FLNA complexes and allows MORs to release to interact with Gs upon subsequent stimulation by morphine. By binding to FLNA, NLX and its analogs prevent this altered MOR–FLNA interaction, thereby preventing the release from the complexes and the resultant altered coupling. There are multiple signaling consequences of the switch to Gs coupling by MORs chronically exposed to opioids, and each may contribute differently to the various behavioral effects of long-term opioid administration such as analgesic tolerance, physical dependence and the possibility of addiction. This notion may explain the multiple beneficial effects of ultra-low-dose opioid antagonist co-treatment, shown to preserve the normal G protein coupling profile of MOR [4]. By identifying the target and binding site of ultra-low-dose NLX and naltrexone, we further elucidate their mechanism of action when combined with opioids. Finally, these findings create an opportunity to formulate a new generation of pain therapeutics that may provide long-lasting analgesia with minimal tolerance, dependence and addictive properties.

## Methods

### Animals

Male Sprague Dawley rats (200-250 g) purchased from Taconic (Germantown, NY) were housed two per cage and maintained on a regular 12-hr light/dark cycle in a climate-controlled room with food and water available *ad libitum.* For identification of NLX-binding protein in MOR immunoprecipitates, four groups of 4 rats were treated twice daily for 7 days with vehicle, NLX (10 ng/kg, s.c.), morphine (10 mg/kg, s.c.), or morphine+NLX. These animals were sacrificed by decapitation 16 hr after the last injection, and whole striatum was harvested on ice immediately. For organotypic striatal slice cultures, brain slices harvested from treatment-naïve rats were maintained and treated *in vitro* as described below. All procedures in this protocol are in compliance with the City College of New York IACUC on the use and care of animals.

### Identification of FLNA in MOR immunoprecipitates

Neuronal membranes (200 µg) were prepared as described previously [4], [25] from striata of rats treated as described above. Membranes were incubated with 1 µM morphine for 5 min at 37°C in Kreb's Ringer solution before solubilization in immunoprecipitation buffer (25 mM HEPES, pH 7.5; 200 mM NaCl, 2 mM MgCl_2_, 1 mM EDTA, 0.2% 2-mercaptoethanol, 50 µg/ml leupeptin, 25 µg/ml pepstatin A, 0.01 U/ml soybean trypsin inhibitor, 0.04 mM phenylmethylsulfonyl floride [PMSF]) containing 0.5% digitonin, 0.2% sodium cholate and 0.5% NP-40 at 4°C with end-over-end shaking for 60 min. The supernatant was collected after centrifugation at 50,000 X g for 5 min to remove insoluble debris before immunoprecipitation. MOR and its associated scaffolding proteins and G proteins were immunopurified together using anti-Gαs/olf or -Gαo antibodies that were immobilized to prevent interference from immunoglobulins. Anti-Gα antibodies (Santa Cruz Biotechnology, Santa Cruz, CA) were covalently cross-linked to protein A conjugated resin in a Seize-X protein A immunoprecipitation kit (Pierce-ENDOGEN, Rockford, IL) according to manufacturer's instructions. MOR-G protein-scaffolding protein complexes in solubilized brain lysate were first isolated by immunoprecipitation in which 200 µg solubilized brain membrane extract from striatum was incubated with immobilized anti-Gα-protein A-resin at 4°C overnight. After centrifugation and three washes with phosphate-free Kreb's-Ringer (pH 7.4) containing mixtures of protease and protein phosphatase inhibitors at 4°C, the MOR-G protein-scaffolding protein complexes were eluted with 200 µl of neutral pH gentle antigen elution buffer, diluted 5-fold with immunoprecipitation buffer, and immunoprecipitated with anti-MOR at 4°C for 4 hr followed by 50 µl protein A/G-conjugated beads (Santa Cruz Biotechnology) for 2 hr. The immunoprecipitates containing MOR-G protein-scaffolding protein complexes were collected by centrifugation and washed twice with phosphate-free Kreb's-Ringer. The washed immunocomplex was re-suspended in 75 µl phosphate-free Kreb's-Ringer and solubilized by combining with 75 µl of 2X PAGE sample preparation buffer (62.5 mM Tris-HCl, pH6.8; 20% glycerol, 4% SDS; 10% 2-mercaptoethanol, 0.1% bromophenol blue) and boiled for 5 min. The levels of selective MOR-associated scaffolding proteins were determined by Western blotting using specific antibodies directed against various cytoskeletal and scaffolding proteins including FLNA, MAP1B and yaotio.

### NLX binding to FLNA-expressing cells

To confirm FLNA as the high-affinity target of NLX, we assessed [^3^H]NLX binding to the human melanoma cell line M2 subclone that was stably transfected with human filamin A cDNA (obtained from Drs. Stossel and Ohta at Harvard Medical School). Membranes prepared from A7 cells (100 µg) were incubated in binding medium (50 mM Tris HCl, pH7.5; 100 mM NaCl; and protease and protein phosphatase inhibitors) with 500 pM [^3^H]NLX in the presence of 10 µM of either morphine or NTX at 37°C for 30 min. Total incubation volumes were 500 µl. Non-specific binding was defined by 1 µM NTX. Membranes prepared from the parent M2 cells (200 µg) that do not express FLNA served as a negative control for [^3^H]NLX binding, and A7 cell membranes (200 µg) incubated with 2 nM [^3^H]DAMGO illustrated the lack of MOR in both cell lines. Reactions were terminated by rapid filtration through 3% BSA-treated GF/B membranes under vacuum. Filters were washed twice with 5 ml ice-cold binding medium, and [^3^H]NLX retained on the filters was measured by liquid scintillation spectrometry.

In a separate experimental series, whole cell binding of [^3^H]NLX in intact A7 and M2 was performed. A7 and M2 cells were grown on 35-mm dishes until 80% confluent. After two washes with PBS (37°C), [^3^H]NLX (0.5 nM) was added to cells and incubated for 30 min at 37°C in the absence or presence of 10 µM pentapeptide FLNA fragment, VAKGL. Following removal of [^3^H]NLX containing binding medium, cells were washed twice with PBS (37°C), collected and [^3^H]NLX in cells were counted by scintillation spectrometry.

To visualize NLX binding, A7 and M2 cells were grown on chambered slides (Nalge Nunc, Naperville, IL) to 80% confluency. FITC-NLX (10 nM, Invitrogen) was added to the cells in 0.5% FBS-containing culture medium and incubated for 30 min at 37°C in the presence or absence of 10 µM VAKGL or VAAKGL. Following incubation, medium was removed and cells were washed three times with warm PBS. Cells were then fixed in 10% formalin-PBS overnight at 4°C and coverslipped. The bound FITC-NLX was visualized with a fluorescence microscope.

### Affinity measurement

A competition (displacement) curve was generated for the inhibition of [^3^H]NLX binding by naltrexone to membranes prepared as described above from FLNA-expressing A7 cells. A nonlinear curve-fit analysis was performed using competition equation that assumed two saturable sites for naltrexone curve comprising of 16 concentrations ranging from 0.1 pM to 1 µM. Six experiments each using a different set of A7 cells were included in the analysis.

### Determination of binding site using FLNA peptides

To determine the NLX binding site on FLNA, various overlapping peptides encoding the c-terminal section of FLNA were used to compete for [^3^H]NLX binding to FLNA using either A7 cell membranes or purified FLNA from A7 or SK-N-MC cells. Peptides were generated by Sigma-Genosys (The Woodlands, TX). The reaction mixture consisted of 100 µg A7 membranes or 2 µg purified FLNA, 500 pM [^3^H]NLX, and 10 µM of either FLNA_2550–2560_, FLNA_2556–2565_, FLNA_2561–2570_, FLNA_2566–2575_ or FLNA_2576–2581_ in 500 µl binding medium. With FLNA purified from SK-N-MC cells, 1 µM of the irreversible MOR antagonist β-funaltrexamine (β-FNA) was used to demonstrate binding independent of MOR. The reactions were carried out at 37°C for 30 min and terminated by rapid filtration through 3% BSA-treated GF/B membranes under vacuum. Filters were washed twice with 5 ml ice-cold binding medium, and [^3^H]NLX retained on the filters was measured by liquid scintillation spectrometry.

### Alanine scan of pentapeptide on FLNA binding

To determine the essential amino acid(s) within the NLX-interacting pentapeptide, four additional pentapeptides, each with one amino acid replaced by alanine, were used along with the correct FLNA_2561-2565_ pentapeptide to compete for [^3^H]NLX binding to FLNA using A7 cell membranes. Peptides were generated by Sigma-Genosys. The reaction mixture consisted of 500 pM [^3^H]NLX, 200 µg A7 membranes, and 10 µM pentapeptide (AAKGL, VAKGL, VAAGL, VAKAL or VAKGA) in 500 µl binding medium. Reactions were conducted at 37°C for 30 min and terminated by rapid filtration through 3% BSA-treated GF/B membranes under vacuum. Filters were washed twice with 5 ml ice-cold binding medium, and [^3^H]NLX retained on the filters was measured by liquid scintillation spectrometry.

### Organotypic striatal slice cultures

In this set of experiments, rat brain slice organotypic culture methods were modified from those published previously [26], [27]. Striatal slices (200 µM thickness) were prepared using a McIlwain tissue chopper (Mickle Laboratory Engineering Co., Surrey, UK). Slices were carefully transferred to sterile, porous culture inserts (0.4 µm, Millicell-CM) using the rear end of a glass Pasteur pipette. Each culture insert unit contained 2 slices and was placed into one well of the 12-well culture tray. Each well contained 1.5 ml of culture medium composed of 50% MEM with Earl's salts, 2 mM L-glutamine, 25% Earl's balanced salt solution, 6.5 g/l D-glucose, 20% fetal bovine serum, 5% horse serum, 25 mM HEPES buffer, 50 mg/ml streptomycin and 50 mg/ml penicillin. The pH was adjusted to 7.2 with HEPES buffer. Cultures were first incubated for 2 days to minimize the impact of injury from slice preparation. Incubator settings throughout the experiment were 36°C with 5% CO_2_.

To induce tolerance, culture medium was removed and the culture insert containing the slices was gently rinsed twice with warm (37°C) phosphate-buffered saline (pH 7.2) before incubation in 0.1% fetal bovine serum-containing culture medium with 100 µM morphine for 1 hr twice daily (at 9–10 AM and 3–4 PM) for 7 days. To assess the effect of ultra-low-dose of NLX on the chronic morphine-induced signaling switch, some slices were exposed to 100 µM morphine plus 10 pM NLX. To determine whether NLX's protective effect occurs by binding to FLNA at FLNA_2561–2565_, slices were incubated with morphine plus NLX with the addition of 10 µM FLNA_2550–2560_, FLNA_2561–2570_, or FLNA_2566–2575_. Slices were returned to culture medium with normal serum after each drug exposure. Tissues were harvested 16 hr after the last drug exposure by centrifugation.

### MOR–Gs coupling in slice cultures

For determination of MOR–G protein coupling, slices were homogenized to generate neuronal membranes. Membranes (400 µg), prepared as described above, were incubated with either 1 µM morphine or Kreb's-Ringer solution for 10 min before solubilization in 250 µl of immunoprecipitation buffer (25 mM HEPES, pH7.5; 200 mM NaCl, 1 mM EDTA, 50 µg/ml leupeptin, 10 µg/ml aprotinin, 2 µg/ml soybean trypsin inhibitor, 0.04 mM PMSF and mixture of protein phosphatase inhibitors). Following centrifugation, striatal membrane lysates were immunoprecipitated with immobilized anti-Gαs/olf or -Gαo conjugated with immobilized protein G-agarose beads. The level of MOR in anti-Gαs/olf or -Gαo immunoprecipitates was determined by Western blotting using specific anti-MOR antibodies.

### cAMP accumulation in slice cultures

To measure the magnitude of MOR-mediated inhibition of cAMP production, brain slices were incubated with Kreb's-Ringer (basal), 1 µM DAMGO, 1 µM forskolin or 1 µM DAMGO+1 µM forskolin for 10 min at 37°C in the presence of 100 µM of the phosphodiesterase inhibitor IBMX. Tissues were homogenized by sonication and protein precipitated with 1M TCA. The supernatant obtained after centrifugation was neutralized using 50 mM Tris, pH 9.0. The level of cAMP in the brain lysate was measured by a cAMP assay kit (PerkinElmer Life Science, Boston, MA) according to manufacturer's instructions.

### Data analysis

All data are presented as mean±standard error of the mean. Treatment effects were evaluated by two-way ANOVA followed by Newman-Keul's test for multiple comparisons. A two-tailed Student's *t* test was used for *post hoc* pairwise comparisons. Data are presented as means±s.e.m. The threshold for significance was p<0.05.
